The article "Uterine salvage management for atonic postpartum hemorrhage using “modified lynch suture”" was retracted in 2025. Reasons: unreliable results or conclusions; lack of ethics approval or compliance.

# Uterine salvage management for atonic postpartum hemorrhage using “modified lynch suture”

**DOI:** 10.1186/s12884-016-1000-2

**Published:** 2016-08-27

**Authors:** M. El-Sokkary, K. Wahba, Y. El-Shahawy

**Affiliations:** Dept. of Obstetrics and Gynecology (OBGY), Ain Shams University Maternity Hospital, Cairo, Egypt

**Keywords:** Postpartum hemorrhage, Atony, B-Lynch, Uterine salvages

## Abstract

**Background:**

To assess the effectiveness of the new modified technique in order to control bleeding in women presenting with atonic, flabby uterus compared to the most commonly described technique of classic B-Lynch suture.

**Method:**

This study included 160 women of uncontrolled atonic postpartum hemorrhage delivered by cesarean section at Ain Shams University Maternity Hospital between January 2013 and October 2015. Participants were randomly assigned following simple randomization procedures (computerized random numbers) and divided into two groups. Group, I (80 patients) operated upon by the modified (new technique) stitch while group II (80 patients) operated upon by the classic technique. The ultimate goals were to stop blood loss after placement of the sutures and avoid life-saving hysterectomy thus preserving the life and fertility of the patient.

**Results:**

The modified new technique was done in 80 patients with atonic postpartum hemorrhage and it was found to be superior to the classic technique with a success rate 95 % (4 cases needed hysterectomy as a lifesaving measure) compared to 85 % with the classic technique (in 12 cases, a life-saving hysterectomy was done).

**Conclusions:**

This technique can replace the classic B-lynch in flabby unresponsive atonic uteri as it has 8 shaped placement of the stitch which causes more firm compression on the uterus and simultaneous bilateral uterine artery ligation. This technique was proved valuable and successful in many patients who suffer from uncontrolled massive postpartum hemorrhage (PPH).

## Background

Primary postpartum hemorrhage (PPH) refers to the bleeding from the genital tract that is more than 500 ml after vaginal delivery or more than 1000 ml following cesarean section during the first 24 h following delivery of the fetus [1]. However, intraoperative blood loss estimation is inaccurate in most cases; therefore, the American College of Obstetrics and Gynecology has defined it as a drop of hematocrit value of more than 10 % from the predelivery value [2]. PPH accounts for most cases of maternal morbidity and mortality in developing countries [3]. The causes of PPH include trauma, retained placenta, abnormal coagulation that may be congenital or acquired, and atonic uterus, which is one of the preventable causes of primary PPH and accounts for more than 80 % of cases of primary PPH [4].

The article "Uterine salvage management for atonic postpartum hemorrhage using “modified lynch suture”" was retracted in 2025. Reasons: unreliable results or conclusions; lack of ethics approval or compliance.

In March 1997, Lynch [5] published his brace suture for controlling PPH when other primary measures failed. The procedure was simple and effective with the primary goal to compress the uterus without occluding the uterine arteries or uterine cavity [5]. Since this publication, more than 10 variants of uterine compressing sutured have been reported [6–10]. If this method fails, the next step will be vascular ligation (uterine, ovarian and hypogastric) or hysterectomy as a last resort [5]. In the current literature, a new modified technique of classic B-Lynch has been reported that has more effective compression on the uterus with added hemostatic effect of uterine artery ligation.

## Method

This prospective clinical trial was performed in the Department of Obstetrics and Gynecology, Ain Shams University Maternity Hospital, Cairo, Egypt, between January 2013 and October 2015. A total of 160 women who suffered from PPH during lower segment cesarean section (LSCS) and were not responding to uterotonics were operated upon by the modified technique or the classic one after counseling of the patient and a written consent given by the patient.

### Patient groups

160 women with PPH refractory to uterotonics were divided into:

- **Group I** (modified technique): 80 patients were operated upon by the new technique
- **Group II** (classic technique): 80 cases were operated upon by the classical technique of B-Lynch.

### Patient selection

Patients under general anesthesia with atonic postpartum hemorrhage refractory to uterine massage, ecbolics (oxytocin 30 units IM, methergine 0.25 mg, misoprostol 1000 μg rectal) and bimanual compression. If these measures failed, the modified or classic technique was done randomly. 5 min later, the patient is observed abdominally and vaginally for bleeding. If bleeding had stopped, closure of the abdomen with intraperitoneal drain is done, but if bleeding still continued, this represents a failure of the compression sutures thus, internal iliac artery ligation or hysterectomy will be done.

### Exclusion criteria

Patients with traumatic PPH, DIC, bleeding diathesis, retained parts of the placenta or cases with uterine anomalies.

### Outcome

- Successful: if the bleeding stopped and no need for hysterectomy
- Unsuccessful: if the bleeding continued and there is a need for hysterectomy

### Randomization

For allocation of the participants, a computer-generated list of random numbers was used and was kept in Ain Shams Maternity Hospital computer and with research supervisors. Participants were randomly assigned for following simple randomization procedures (computerized random numbers) to 2 treatment groups modified Lynch and classical Lynch groups. Group assignments were allocated according to a computer-generated randomized series, were kept in sealed envelopes.

The article "Uterine salvage management for atonic postpartum hemorrhage using “modified lynch suture”" was retracted in 2025. Reasons: unreliable results or conclusions; lack of ethics approval or compliance.

### Postoperative results

Vital data, urine output, follow up of any vaginal bleeding, the output of the intraperitoneal drains, hemoglobin and hematocrit concentration. Blood transfusion was given according to patient preoperative hemoglobin and amount of blood loss intraoperative.

In stable cases, observations were made for 48 h, then discharging the patient with discharge card, including all the operative details to be rechecked after one week for any abnormality (wound gaping, deep venous thrombosis, puerperal sepsis, uterine wall necrosis, vesicovaginal fistula).

### Steps of the new modified Lynch technique (See fig. 1)

Exteriorize the uterus, removal of sutures of lower segment cesarean section. The assistant stretched up the uterus, the 1st stitch is placed 2 cm below the lower segment incision and 2 cm medial to the lateral angle to come on the same side on the upper flap then cross on the fundus to the contralateral side above the uterosacral then to the other uterosacral then to the contralateral flap in a figure of eight fashion then after tightening of this suture the needle is passed through avascular area in the broad ligament to the back while the tape is passed through a window on the opposite side made by an artery forceps to become on the posterior aspect of the uterus. Tightening of the transverse suture is done.

**Fig. 1:** Steps of the new modified Lynch technique

### Advantages of the modified technique over the classical technique

The 8 shaped ligatures appear to be more hemostatic and compressing the uterus. Also, the transverse limb ligates the uterine artery with more compression on the lower segment, so it is more effective in case of placenta previa or bleeding from the lower segment in general.

## Results

A total of 160 women was recruited in the current study. The clinic-epidemiological data of women under the study were analyzed, in group I, the mean age was 29.6 ± 4.5 years, the mean parity was 1.55 ± 1.35, the mean weight was 76 ± 13.13151 kg, the gestational age was 39.1 ± 1.1 weeks and the neonatal birth weight was 3.49 ± 0.365 kg compared to group II in whom the mean age was 29.3 ± 5.1 years, the mean parity was 1.6 ± 1.21, the mean weight was 79 ± 12.325 kg, the gestational age was 38.7 ± 1.8 weeks and the neonatal birth weight was 3.49 ± 0.365 kg with no significant difference between the two groups (*P* < 0.001). The modified new technique was done in 80 patients with atonic postpartum hemorrhage refractory to usual measures and it was found to be superior to the classic technique with a success rate 95 % (4 cases needed hysterectomy as a lifesaving measure) compared to 85 % with the classic technique (in 12 cases, a life-saving hysterectomy was done) as shown in Table 1.

The article "Uterine salvage management for atonic postpartum hemorrhage using “modified lynch suture”" was retracted in 2025. Reasons: unreliable results or conclusions; lack of ethics approval or compliance.

**Table 1:** Shows the clinic-epidemiological, operative and postoperative data of women under the study

Parameter	G1	G2	*P*-value
Age (year) Mean ± SD	29.6 ± 4.5	29.3 ± 5.1	0.694
Parity	1.55 ± 1.35	1.61 ± 1.21	0.431
Weight	76 ± 13.151	79 ± 12.325	0.139
Gestational age	39.1 ± 1.1	38.7 ± 1.8	0.092
Neonatal birth weight	3.496 ± 0.365	3.397 ± 0.389	0.099
Postoperative blood loss	324 ± 105	568 ± 209	0.0001 (HS)
Need for blood transfusion	2.8 ± 0.5	4.2 ± 0.8	0.0001 (HS)
Need for hysterectomy	4	12	0.0001 (HS)
Hospital stay	2.8 ± 1.5	2.7 ± 1.6	0.684
Duration of procedure	6 ± 0.95	3 ± 1.3	0.0001 (HS)
Pre-operative Hb%	9.8 ± 1.2	10.1 ± 1.3	0.131
Post-operative Hb%	8.7 ± 1.1	8.9 ± 1.8	0.398
Bleeding from multiple bites	7	13	0.152
Hematometra	1	5	0.212
Wound hematoma	4	4	1.00
Wound infection	4	4	1.00
Fever	5	8	0.563

Table (1) shows that there was no significant difference between the two groups as regards the clinic-epidemiological characters of the study groups and the postoperative data, but the modified new technique was found to be superior to the classic technique with a success rate 95 % compared to 85 % with the classic technique

The two groups were compared as regards the complications of the conservative operative intervention, as regards the bleeding from multiple bites; it was clear that it was lower in group I when compared to group II which appears due to the hemostatic added effect of uterine artery ligation but the difference was not statistically significant, the same with the other postoperative parameters as development of hematometra, wound infection or post-operative fever, there was no significant difference between the two groups (Table 1).

## Discussion

Postpartum hemorrhage is a potentially life-threatening complication of fetal delivery [11]. It may occur after vaginal delivery (4 %) or caesarean births (6 %) [12, 13]. The most important step in the management of PPH is to identify and correct the underlying cause [14]. Most of the cases of PPH can be controlled by traditional treatment modalities like uterotonics, uterine massage, bimanual compression and balloon tamponade [14]. Uncontrolled PPH is usually managed by different uterine suture techniques (modified B-Lynch, and square suture) or with stepwise devascularization surgical procedures. These techniques have reported variable outcomes and many of the patients finally require emergency hysterectomy [5, 7, 14]. A review of peripartum or cesarean hysterectomy reported an average mortality rate of 4.8 % [15]. This does not mean that hysterectomy caused this high maternal mortality, but critically ill situations requiring this surgery may eventually cause it. Indeed, cesarean hysterectomy is one of the most difficult obstetric surgeries and is always challenging [16]. The surgical method of controlling uterine bleeding by inserting B-Lynch suture has been developed to reduce the incidence of emergency hysterectomy and to preserve fertility in these patients. Because of simplicity of application and less time taken to put the modified B-Lynch stitch, it should be the preferred choice [6].

The article "Uterine salvage management for atonic postpartum hemorrhage using “modified lynch suture”" was retracted in 2025. Reasons: unreliable results or conclusions; lack of ethics approval or compliance.

### Various parameters in the current study are compared as follows

In Khatoon et al. study [17], B-Lynch stitch was applied in 9 cases, i.e. 60 % after vaginal delivery and on 6 cases i.e. 40 % during cesarean section. In the current study the new technique of the B-Lynch stitch was taken on 160 cases during cesarean section, but actually, in our institute the new technique is now being performed on cases also after vaginal delivery and on the closed uterus to avoid the additional bleeding on incision of the uterus but this is still under trial.

In a prospective study of Hackenthal et al. [18], Hb difference is 3gm% after using the modified B-Lynch technique and in the current study, the mean intraoperative blood loss was 568 ± 209 ml after classical technique and 324 ± 105 ml after the new technique with a highly significant difference between the two groups. After the blood transfusion according to the clinical condition, there was no significant difference between the two groups as regards the postoperative hemoglobin.

In Koh et al. study [19], 4 patients required more than 3 units of blood transfusion and 2 patients did not require any blood transfusion while in the current study the mean units of blood required was 4.2 ± 0.8 in the group who was operated upon by the classical technique and was 2.8 ± 0.5 in the group who was operated upon by the new technique with highly significant difference between the two groups, reflecting the effectiveness of new modified B-Lynch stitch in the control of atonic postpartum hemorrhage.

In a study of Anamika et al. [20], time was taken to put stitch was 11 to 20 min in 35 patients and less than 10 min in 3 patients, more than 20 min in 5 patients. In Our study, time taken to put stitch of the classic technique was 3 ± 1.3 while the time taken to put stitches of the new technique was 6 ± 0.95 with highly significant difference between the two groups, but this factor may be changed with more training and familiarity with the new technique and must be kept in mind the effectiveness of the new method.

The article "Uterine salvage management for atonic postpartum hemorrhage using “modified lynch suture”" was retracted in 2025. Reasons: unreliable results or conclusions; lack of ethics approval or compliance.

Study conducted by Hackenthal et al. [18] and Anamika et al. [20] had a success rate of 100 %, thus proving that this technique was highly effective and 1 patient died on the 21st postpartum day due to Acute Respiratory Distress Syndrome and Septicaemia In Our study success rate was 85 % with the classic technique and 95 % with the new technique with highly significant difference between the two groups with no mortalities..

In a prospective study conducted by Ghodake et al. [21], 31 patients underwent B-Lynch stitch, out of which 5 patients had a post-operative fever, 3 patients had surgical wound gaping. In our study, 8 patients had a post-operative pyrexia in the group operated upon by the classic technique and 5 patients in the group operated upon by the new technique with a highly significant difference between the two groups. But as regards wound infection and gaping there was no significant difference between the two groups. In Our study, there were no major complications.

## Conclusion

The new technique of the B-Lynch is highly effective in controlling an atonic postpartum hemorrhage so we suggest strongly this technique as an alternative safe option to stop an atonic postpartum hemorrhage. There was no adverse effect on the fertility potential for the observed 2 years; however, a long-term follow-up is required to comment on its actual rate.

All pertinent study information was explained to them and they were informed that rejection or withdrawal from the study will not affect any medical service provided. A summarized study information sheet was shown to all cases before obtaining their verbal agreement. Finally, an informed verbal consent was obtained and witnessed by the attending nurse. A log book was created including the participant’s study number and the date of consent. The IRB waived the requirement for taking a written consent as the research had minimal risk of harm to subjects and involved no risky procedures for which written consent is required.
